# Analysis of the Clinical Effect of Implementing Health Education in the Process of Ministration Elderly Hypertensive Sufferers

This article has been retracted.

**DOI:** 10.1155/2022/8357617

**Published:** 2022-09-13

**Authors:** Xin Yu, Hui Lyu, Bo Yu, Xueling Xu, Yi Xu

**Affiliations:** ^1^Health Management Center, The First Affiliated Hospital of Dalian Medical University, Dalian 116011, China; ^2^Intensive Care Unit, The Second Hospital of Dalian Medical University, Dalian 116027, China; ^3^Emergency Ward, The Second Hospital of Dalian Medical University, Dalian 116027, China

## Abstract

The clinical effect of implementing health education in ministration elderly hypertensive sufferers is analyzed. Two hundred hypertensive sufferers admitted to our hospital from February 2020 to April 2021 are selected. The two sets of sufferers are randomly divided into the examination set and the control set using the random number table method, with 100 cases in each set. The control set is given routine ministration care, and the examination set is given routine ministration to implement health education; these indicators include: the blood pressure control compliance, Self-rating Anxiety Scale (SAS), Self-rating Depression Scale (SDS), and the Chinese version of Perceived Stress Scale (CPSS) scores; the compliance rate of health knowledge score, serum Angiotensin II (Ang II), Endothelin-1 (ET-1) and Superoxide Dismutase (SOD) standards, medication compliance, prognosis quality of life, and cumulative occurrence of MACCE are compared. The experimental results show that the application of health education in the ministration process of elderly hypertensive sufferers can effectively enhance the blood pressure of the sufferers, reduce the negative emotions and psychological pressure of the sufferers, enhance the quality of life of the sufferers, and reduce the prognosis of recurrence and the occurrence of adverse cardiovascular events.

## 1. Introduction

With the development of the economy and the enhancement of people's living standards, the prevalence of cardiovascular and cerebrovascular ailments such as hypertension, diabetes, and hyperlipidemia is increasing year by year, especially in the elderly, which has a serious impact on the prognosis of elderly sufferers [1]. Hypertensive sufferers have low awareness, low control ability, and low therapy rate. Therefore, it is urgent to enhance the blood pressure control standard of sufferers [2]. In addition to medication, health education and exercise therapy also support blood pressure control. Due to the growing health needs of sufferers, the conventional health education model is relatively simple and the intervention effect is limited, so the health education model is a new trend in clinical development [3, 4]. Previous studies have found that physical intervention for hypertensive sufferers has obvious antihypertensive effects, especially that health education is suitable for most hypertensive sufferers, but there are certain disparities in the physical conditions of different individuals, and individualized health education programs can reduce the risk. At the same time, the impact effect is maximized [5–7].

In order to enhance their health behaviors and reduce psychological stress, this examination carried out health education for elderly hypertensive sufferers, and further enhance blood pressure standards. The examination selected 200 hypertensive sufferers admitted to our hospital from February 2020 to April 2021. In the study, the two sets of sufferers are randomly divided into the examination set and the control set. The experimental results show that the application of health education in the ministration process of elderly hypertensive sufferers can effectively enhance the blood pressure of the sufferers, reduce the negative emotions and psychological pressure of the sufferers, enhance the quality of life of the sufferers, and reduce the prognosis of recurrence and the occurrence of adverse cardiovascular events.

The rest of this paper is organized as follows: Section 2 discusses related work, followed by the sufferers' information and examination methods designed in Section 3.  Section 4 shows the experimental results and analysis, and Section 5 is the conclusion, which summarizes and looks forward to the prospects for health education in ministration elderly hypertensive sufferers.

## 2. Related Work

Hypertension is one of the chronic ailments with the extensive number of sufferers in my country, but the awareness rate, therapy rate, and control rate are still at a low standard. In order to enhance the prevention and control of hypertension, health information publicity, drug therapy, psychological counseling, and dietary guidance should be strengthened, along with exercise interventions and other measures [8, 9]. The application of health education in ministration in this examination starts from the sufferer's cognition, attitude, and psychology, enhances the sufferer's cognition and enthusiasm for therapy, then disseminates hypertension-related knowledge through publicity materials, bulletin boards, lectures, etc [10]., and finally strengthens drug use/diet/life guidance to gradually achieve the purpose of health education [11, 12]; in addition, health education is used in ministration to arrange an appropriate amount of exercise intensity for sufferers according to the sufferer's oxygen uptake test, and to ensure the effect of exercise intervention while taking into account the actual situation of the sufferer. The results of the examination showed that after 3 months, 6 months, and 12 months of the intervention in the two sets, the blood pressure control rate and the compliance rate of the sufferers in the examination set were notoriously higher than those in the control set, both (*P* < 0.05), indicating that the application of health education in ministration can enhance the sufferers' blood pressure, i.e., has an antihypertensive effect.

Relevant studies have pointed out that ideal health behaviors (including non-smoking, reasonable diet, weight control, and exercise compliance) are independent protective factors for isolated diastolic hypertension, indicating that the application of health education in ministration can not only reduce the risk of hypertension, but also increase the risk of hypertension[13]. The results of this examination showed that after ministration, the Self-rating Anxiety Scale (SAS), Self-rating Depression Scale (SDS), and the Chinese version of Perceived Stress Scale (CPSS) scores of the two sets of sufferers were notoriously enhanced, and the enhancement effect of the examination set was notoriously better than that of the control set (*P* < 0.05). The scores and the compliance rate were notoriously enhanced, and the enhancement effect of the examination set was notoriously better than that of the control set (*P* < 0.05), suggesting that diversified health education combined with individualized aerobic exercise can promote the healthy behavior of sufferers. Decomposition of the reasons is related to the promotion and supervision of health knowledge in the application of health education in ministration, and the aerobic exercise promoted in education takes into account the disparity in individual physical fitness, and formulates a suitable exercise intensity for each person to ensure effective completion [14]. In recent years, studies have found that in addition to genetic factors and environmental factors, psychological stress can also induce the development of hypertension. This is because stress can affect the balance of the body. When it exceeds the body's ability to regulate, some pathological changes will occur, which will eventually lead to the development of hypertension. In addition, the application of health education in ministration can reduce the psychological pressure of sufferers [15]. Many clinical studies have shown that cognitive behavioral intervention can effectively reduce the psychological pressure of sufferers, reduce the impact of negative emotions, and contribute to the smooth development of therapy and intervention. The application of health education in ministration can introduce hypertension-related knowledge to sufferers from various aspects, which can notoriously enhance the sufferer's cognition. Coupled with targeted psychological counseling, it can reduce the sufferer's pressure emotionally, and aerobic exercise can also enhance the physical and mental health of the sufferer, to release the pressure [16].

In addition, this examination found that after completing the corresponding ministration care, the medication compliance of the examination set was 95.00%, which was notoriously higher than that of the control set (75.00%) (*P* < 0.05); the examination set was notoriously higher than the control set (*P* < 0.05); the main reason for the decomposition is that the application of health education in ministration is based on the theory of knowledge, belief, and behavior, which enhances the standard of knowledge and belief. It can promote individuals to choose a positive attitude to benefit health, and gradually establish a healthy lifestyle. Based on the theory of “Knowledge, Belief and Action,” this examination uses health education in ministration to intervene sufferers. Through the “education” link, sufferers are given ailment-related knowledge guidance to make them clear about the importance of a healthy lifestyle and gain more knowledge, answer sufferers' confusion, and correct their misunderstandings through online Q&A [17, 18]. Endothelin-1 (ET-1) is an active substance produced by ET, which can regulate the contraction of vascular smooth muscle and promote the proliferation and hypertrophy of blood vessels; superoxide dismutase (SOD) is an antioxidant substance produced during aerobic exercise, which is related to bodily functions [19]. This examination found that after ministration, the serum AngII, ET-1, and SOD levels of the two sets of sufferers were notoriously enhanced, and the enhancement effect of the examination set was notoriously better than that of the control set (*P* < 0.05). The expression of serum angiotensin II (Ang II) and ET subjoined the expression of SOD. The possible mechanism of action is as follows: the application of health education in ministration enhances physical function by increasing the content and activity of antioxidant substances, thereby preventing blood pressure from rising; the application of health education in ministration can activate various systems, and increase the secretion of vasodilatory substances. It can reduce the production of vasoconstrictive substances such as Ang II and ET-1, reduce blood pressure, and reduce the incidence of elevated blood pressure and MACCE in prognosis [20, 21].

## 3. Sufferers' Information and Examination Methods

### 3.1. Sufferers' Information

In this examination, 200 hypertensive sufferers admitted to our hospital from February 2020 to April 2021 are selected for the examination, and the two sets of sufferers are randomly divided into the examination set and the control set using the random number table method, with 100 cases in each set. In the examination set, there are 66 males and 44 females; age 55–77 years, mean (65.40 ± 4.82) years old; ailment duration 1–10 years, mean (5.53 ± 0.86) years; and 39 sufferers with hypertension grade I and 61 sufferers with grade II. The control set had 65 males and 45 females; age 55–78 years, mean (64.82 ± 4.78)years; course of ailment 1–10 years, mean (5.44 ± 0.96) years; and 38 sufferers with hypertension grade I and 62 in grade II. The clinical general data such as age and gender are contrasted between the two sets, *P* > 0.05, and there is no extensive disparity between the two sets. All sufferers included in the examination signed the informed consent form. The therapy methods and detection methods used in this examination are all known safe methods in the clinic; the general information and clinical data collected in this examination are only used for examination decomposition, and not for other purposes. The patients were asked to inform of any discomfort during therapy to the doctor in charge in time to decide the next therapy plan; the entire therapy and observation period is 4 weeks; they were also asked to inform the doctor of their condition changes in time, and to not use it privately during therapy. All other medicines and other therapy for the ailment, if used, were also informed to their physician.

### 3.2. Examination Methods

Both sets of sufferers are taking antihypertensive drugs regularly, while the control set adopted a routine health model. The sufferers are introduced to hypertension-related knowledge, the importance of regular medication, dietary precautions, and the benefits of moderate exercise by distributing brochures and health lectures. Lectures are held once a month in the hospital conference room.

For the examination set, health education in routine ministration is implemented as follows: (1) Cognitive intervention: conduct one-on-one conversations to understand the sufferer's psychological state, cognition of the ailment and coping methods, and provide targeted psychological intervention, including the sufferer explaining the impact of negative emotions on blood pressure, and working with the sufferer. Analyze the reasons for negative emotions and guide them to face the ailment positively. (2) Health propaganda and education: Set up bookshelves and propaganda columns in out-sufferer halls and departments (replaced once a week), and place hypertension propaganda materials for sufferers to read. Every Tuesday afternoon, nurses lead sufferers to read relevant information on hypertension, explain in detail the content on the bulletin board, hold health lectures, and invite senior hypertensive physicians in the hospital to explain the causes of hypertension, therapy plans, usage and dosage of commonly used drugs, and non-compliance with the doctor's advice. The hazards of taking medicines, dietary precautions, non-drug therapy methods, etc., are also explained. (3) Medication/diet/life guidance: For medication, make a small card listing the names, usage, and dosage of commonly used antihypertensive drugs and distribute them to each sufferer, and ask them to tick the names of the drugs they are currently using and carry them with them; secondly, set up a WeChat set to send a message before meals to remind sufferers to take the medicine and the dosage of the medicine, and ask the sufferer to report the medicine situation in the set before going to bed every day. In terms of diet, nurses formulate nutritional recipes and send them to the WeChat set every week. Sufferers choose according to their own preferences and actual conditions. At the same time, they require a low-sodium diet, should quit smoking and drinking, and eat more fruits and vegetables. In terms of life, it is recommended that the sufferers have regular work and rest, moderate exercise, and develop a personalized exercise plan for the sufferer.

Serum Ang II, ET-1, and SOD standards: 5 ml of fasting cubital venous blood is collected from the sufferers before and after intervention, and the supernatant is collected after centrifugation to detect Ang II, ET-1, and SOD content, of which Ang II is detected by radioimmunoassay, SOD is detected by Ding's method, and ET-1 is detected by nitrate reductase method.

### 3.3. Observation Indicators

There are seven observation indicators as follows:

1. Blood pressure control at 3 months, 6 months, and 12 months and blood pressure compliance rate in the two sets are observed;
2. Physiological status scores of the sufferers in the two sets before and after nursing are compared, and SAS, SDS, and CPSS scores designed by our hospital are used; SAS has a total of 20 items, and the scoring standard of each item is 1–4 points. Scores >50 indicate that the sufferers have anxiety tendency, and the higher the score, the higher the sufferer's anxiety degree. SDS has 20 items, and the scoring standard of each item is 1–4 points. A score >53 indicates that the sufferer has depression tendency, and the higher the score, the more serious the depression degree. CPSS consists of three dimensions, with scores ranging from 22 to 110, with higher scores indicating lower pain levels.
3. To observe the health knowledge score and the health behavior score and the standard rate before and after nursing, we used our hospital's hypertension knowledge scale for evaluating the two sets of sufferers with high blood pressure levels of knowledge, a total of 22 items, including 6 dimensions: hypertension criterion (2, 0 ∼ 2), drug therapy (article 4, 0 ∼ 4), adherence (article 4, 0 ∼ 4), lifestyle (5, 0 ∼ 5), food (2, 0–2 points), and complications (5 cases, 0–5 points). Each item is divided into “yes,” “no,” and “do not know,” with 1 point given for each correct answer and 0 point for wrong answers or do not know. The total score ranges from 0 to 22 points, and the higher the score, the better the knowledge level.
4. Serum Ang ii, ET-1, and SOD levels are observed before and after nursing.
5. Analysis of medication compliance before and after nursing is observed in the two sets. The treatment compliance of sufferers in the two sets after nursing management is observed, and the criteria are as follows: self-designed medication compliance questionnaire: whether sufferers forgot to take hypertension drugs; whether the sufferer forgot to take respiratory therapy or inhaled medicine in the past 2 weeks; whether to reduce the drug dose or stop taking the drug when the disease worsens; forgot to take hypertension medication when leaving home for a long time; whether they took any hypertension medication yesterday; does withdrawal occur when perceived symptoms improve? do you feel you are fully compliant with your hypertension medication regimen? do you find it difficult to take medicine on time? The total score is 8 points, and the results are divided into 3 grades: excellent (6–8), good (3–6 points), and poor (1–3 points). The higher the score, the higher the sufferer's medication compliance. The compliance rate is calculated as: (excellent + good)/total number of cases ×100%.
6. To observe the cumulative occurrence of MACCE in the two sets within one year.
7. Sufferers in both sets are followed up for one year to compare the recurrence rate of the sufferers in the two sets. Recurrence rate = number of recurrences/total number of recurrences ×100%.

### 3.4. Statistical Methods

In this examination, all the data are sorted, and a corresponding database is established for it. All databases are entered into SPSS 26.0 for data processing, and the measurement data are tested for normality. The between-set test is *F*, the independent samples *t*-test is used for the data between sets, the paired-samples *t*-test is used for the data within the set, and the Mann-Whitney *U* test is used for non-normality; the rate representation method is *%*, and the test is *χ2*; when *P* < 0.05, the disparity between the data is considered to be statistically extensive.

## 4. Experimental Results and Analysis

### 4.1. Prognosis of Blood Pressure Control and Blood Pressure Compliance Rate in 3 Months, 6 Months, and 12 Months in the Two Sets

Table 1 shows the prognosis of blood pressure control and blood pressure compliance rate in 3 months, 6 months, and 12 months in the two sets of sufferers. It can be seen from Table 1 that the blood pressure control rate and the compliance rate of the sufferers in the examination set are notoriously higher than those in the control set, and the disparity is statistically extensive in all (*P* < 0.05) after 3 months, 6 months, and 12 months of intervention.

### 4.2. Contrast of SAS, SDS, and CPSS Scores before and after Ministration in the Two Sets

Table 2 shows the contrast of SAS, SDS, and CPSS scores before and after ministration in the two sets. In Table 2, ^*∗*^indicates the contrast with before ministration, *P* < 0.05, and the disparity is statistically extensive. It can be observed from Table 2 that there is no extensive disparity in the SAS, SDS, and CPSS scores between the two sets (*P* > 0.05) before ministration; after ministration, the SAS, SDS, and CPSS scores of the two sets are notoriously enhanced, and the enhancement effect of the examination set is notoriously better. In the control set, *P* < 0.05.

### 4.3. Contrast of Health Knowledge, Health Behavior Scores, and Compliance Rate between the Two Sets before and after Ministration

Table 3 shows the contrast of health knowledge, health behavior scores, and compliance rate between the two sets before and after ministration. In Table 3, ^*∗*^ indicates the contrast with before ministration, *P* < 0.05, and the disparity is statistically extensive. It is clearly evident from Table 3 that before ministration, there are no extensive disparity in the health knowledge, health behavior scores, and compliance rate between the two sets of sufferers (*P* > 0.05); after ministration, the health knowledge, health behavior scores, and compliance rate of the two sets of sufferers are notoriously enhanced, and the enhancement effect of the examination set is notoriously better than that of the control set (*P* < 0.05).

### 4.4. Contrast of Serum AngII, ET-1, and SOD Standards between the Two Sets before and after Ministration

Table 4 shows the contrast of serum AngII, ET-1, and SOD levels between the two sets before and after ministration. In Table 4, ^*∗*^indicates the contrast with before ministration, *P* < 0.05, and the disparity is statistically extensive. It can be seen from Table 4 that there are no extensive disparities in serum AngII, ET-1, and SOD levels between the two sets (*P* > 0.05) before ministration; after ministration, the serum AngII, ET-1, and SOD levels of the two sets are notoriously enhanced, and the enhancement effect in the examination set is better than the control set (*P* < 0.05).

### 4.5. Contrast of Medication Compliance after Ministration between the Two Sets

Table 5 shows the contrast of medication compliance after ministration between the two sets. It can be seen from Table 5 that after completing the corresponding ministration care, the medication compliance in the examination set is 95.00%, which is notoriously higher than 75.00% in the control set, and the disparity is statistically extensive (*P* < 0.05).

### 4.6. Contrast of the Cumulative Occurrence of MACCE between the Two Sets within One Year

All sufferers are followed up for one year, and the follow-up date ended in April 2022.  Figure 1 shows the contrast of the cumulative incidence of MACCE between the two sets within one year. It is clearly evident from Figure 1 that the incidence of MACCE in the examination set is 16% (16/100), which is notoriously lower than 56% (56/100) in the control set, and the disparity is statistically extensive (*P* < 0.05).

### 4.7. Cumulative Recurrence Rate in the Two Sets of Sufferers

Figure 2 shows the contrast of cumulative recurrence rates in the two sets within one year. It can be seen from Figure 2 that the cumulative incidence of hypertension in the examination set is 35% (35/100), which is notoriously lower than 76% (76/100) in the control set, and the disparity is statistically extensive (*P* < 0.05) after one-year follow-up.

## 5. Conclusion

The clinical effect of implementing health education in ministration elderly hypertensive sufferers is analyzed. For hypertensive sufferers, the application of health education in the ministration process can effectively enhance the blood pressure of the sufferers, reduce the negative emotions and psychological pressure of the sufferers, enhance the quality of life of the sufferers, and reduce the prognosis of recurrence and adverse cardiovascular ailments. The occurrence of the event is worthy of clinical application.

## Figures and Tables

**Figure 1:** Contrast of the cumulative incidence of MACCE between the two sets within one year.

**Figure 2:** Contrast of cumulative recurrence rates in the two sets within one year.

**Table 1:** Prognosis of blood pressure control and blood pressure compliance rate in 3 months, 6 months, and 12 months in the two sets of sufferers.

Set	3 months after ministration	6 months after ministration	12 months after ministration
Examination set (*n* = 100)	89 (89.00)	85 (85.00)	80 (80.00)
Control set (*n* = 100)	55 (55.00)	52 (52.00)	45 (45.00)
*χ2*	28.671	25.235	26.133
*P*	＜0.001	＜0.001	＜0.001

**Table 2:** Contrast of SAS, SDS, and CPSS scores before and after ministration in the two sets.

Set	CPSS (Minute)		SAS (Minute)		SDS (Minute)	
	Before ministration	After ministration	Before ministration	After ministration	Before ministration	After ministration
Examination set (*n* = 100)	31.64 ± 6.28	50.19 ± 9.58^*∗*^	78.60 ± 4.45	36.08 ± 3.69^*∗*^	77.59 ± 5.39	33.09 ± 3.19^*∗*^
Control set (*n* = 100)	31.40 ± 6.33	34.35 ± 4.96^*∗*^	78.52 ± 4.36	67.24 ± 6.89^*∗*^	77.53 ± 5.23	67.88 ± 4.23^*∗*^
*t*	−0.103	12.506	1.067	43.692	0.377	42.723
*P*	0.918	＜0.001	0.289	＜0.001	0.707	＜0.001

**Table 3:** Contrast of health knowledge, health behavior scores, and compliance rate between the two sets before and after ministration.

Set	Health knowledge/Behavior (Points)		Compliance rate [*n* (%)]	
	Before ministration	After ministration	Before ministration	After ministration
Examination set (*n* = 100)	7.85 ± 1.15	19.52 ± 3.26^*∗*^	35 (35.00)	79 (79.00)^*∗*^
Control set (*n* = 100)	7.92 ± 1.27	10.47 ± 5.02^*∗*^	37 (37.00)	55 (55.00)^*∗*^
*t*	0.563	16.425	0.256	11.528
*P*	0.497	＜0.001	0.079	＜0.001

**Table 4:** Contrast of serum AngII, ET-1, and SOD levels between the two sets before and after ministration.

Set	AngII (ng/L)		ET-1 (*μ*g/ml)		SOD (U/ml)	
	Before ministration	After ministration	Before ministration	After ministration	Before ministration	After ministration
Examination set (*n* = 100)	60.05 ± 5.83	48.96 ± 4.62^*∗*^	75.60 ± 9.61	53.47 ± 7.28^*∗*^	62.95 ± 5.36	81.50 ± 9.77^*∗*^
Control set (*n* = 100)	59.76 ± 5.91	55.34 ± 4.85^*∗*^	75.50 ± 9.50	67.58 ± 7.46^*∗*^	62.73 ± 5.40	70.06 ± 7.03^*∗*^
*t*	0.114	4.693	0.234	4.393	0.025	7.903
*P*	0.910	＜0.001	0.806	＜0.001	0.980	＜0.001

**Table 5:** Contrast of medication compliance after ministration between the two sets.

Set	Therapy compliance [n (%)]			
	Excellent	Good	Disparity	Compliance
Examination set (*n* = 100)	67	28	5	95 (95.00)
Control set (*n* = 100)	40	35	25	75 (75.33)
*X* ^*2*^				11.623
*P*				＜0.001

## Data Availability

The simulation experiment data used to support the findings of this study are available from the corresponding author upon request.
